# Geriatric Workforce Capacity: A Pending Crisis for Nursing Home Residents

**DOI:** 10.3389/fpubh.2013.00024

**Published:** 2013-07-29

**Authors:** Wei-Chen Lee, Ciro V. Sumaya

**Affiliations:** ^1^Department of Health Policy and Management, School of Public Health, Texas A&M Health Science Center, College Station, TX, USA

**Keywords:** geriatric medicine, geriatrician workforce, geriatric psychiatrist, older adults, nursing home

## Abstract

**Introduction:** The nursing home (NH) population in the US has grown to 1.6 million people and is expected to double by 2030. While 88.3% of NH residents are over 65, the elders aged 85 and more have become the principal group. This demographic change has increased the already high rates of chronic diseases and functional disabilities in NH residents.

**Methods:** This study reviewed the supply of geriatricians in addressing the growing healthcare needs of NH residents.

**Results:** English-written articles between 1989 and 2012 were reviewed. Trend data demonstrate that the geriatrician workforce has decreased from 10,270 in 2000 to 8,502 in 2010. Further, the pipeline analysis of physicians projected to receive board certification in geriatrics (and maintain this certification) indicates a worsening of the already insufficient supply of geriatricians for this vulnerable population.

**Conclusion:** Strategies to attract and maintain a geriatrician workforce are imperative to avert a mounting crisis in the geriatric care in NH and, by extension, other living settings.

## Introduction

The expanding population of older adults in the US and worldwide makes a compelling demand for physicians who can care for the elderly in hospital, long-term care facilities, and in the public health contexts of disease prevention/health promotion. Nursing homes (NH) are an essential component of health service settings particularly for the long-term care of elders with significant disease burdens and disabilities. The current NH population of the United States, 1.6 million, is expected to double by the year 2030 (1). Between 1987 and 1996, the proportions of NH residents who were 85 years old and over rose from 49 to 56% for women and from 29 to 33% for men (2). More than two-thirds of NH residents have multiple chronic health problems. Among them, approximately 60% have multiple mental/cognitive diagnoses (3, 4). Further, functional disability of NH residents has also increased. Nearly 72% of NH residents needed help with three or more activities of daily living (*ADLs*) in 1987, and the proportion increased to 83% of residents in 1996 (2). These health problems and worsening functional disability are significantly associated with cost increases exceeding $120 billion per year (5).

As a result of changing demographics in recent times, the needs for NH health care services and public health services are clearly and dramatically increasing (6–8). Yet a number of reports indicate that geriatricians, physician subspecialists educated and trained to provide quality health care services to the older adults, are declining (6, 9). There is also inadequate data monitoring the number and impact of NH physicians including geriatric specialists (10). Not only can geriatricians provide direct health care but they can also serve as supervisors and coordinators of care to the elderly across health disciplines (11–13). Geriatricians could also be valuable resources in working with public health issues in the aging population. The purpose of the study is to make a more current, critical assessment of the increasing health service needs of a rapidly growing aging population residing in NHs and the capacity of the geriatrician workforce to meet these needs. The findings of this study will have implications for quality health services and health of NH residents and, by extension, to the nation’s older adults in other living settings.

## Methods

Articles from 1989 to the 2012 were obtained for review from MEDLINE and PUBMED literature databases. The key words were NH, nursing facility, elderly health care, older adult health care as healthcare consumers, and geriatrician and geriatric-trained physician as healthcare providers. Trend data from serial National NH Surveys (NHHS) were used to reflect complex service demand of NH residents currently and in the future. The studies focused on overall capacity of education and training in geriatric medicine as well as barriers to recruitment and retention of geriatricians were also included. The research regarding non-USA information was excluded. The specific categories of information solicited through the research review were:

(1) Health care consumer (elderly population in NH): trends and characteristics of the NH elderly population such as enumeration, residents’ age, functional status, and utilization of healthcare services;
(2) Health care provider (geriatricians or geriatricians-in-training): trends in enumeration, personal characteristics, and pipeline of future geriatricians available to provide personal health and public health services to NH residents.

## Results

Seventy-seven published studies covering the special categories listed above were included for review and analysis. All the studies chosen were national in scope; 73 (94.8%) were published after 1999. Studies variably provided serially published data covering a number of years and able to yield longer term trend information.

### Healthcare consumer: Older adult/nursing homes

#### Aging population trend

Data released in 1990 and 2000 by the U.S. *Census Bureau* indicated that the number of the nation’s aging population (65 years and older) is the fastest growing segment of the entire population (14–16). Eighteen million people (6.54% of total population) were 65–74 years old in 1990; more than double of the number was projected by 2030 (40.11 million). The number of people between 75 and 84 years old in 2050 is projected to equal 2.4 times the number in 1990. For the population 85 years and older, there were 4.24 million in 1990 (1.51% of total population) and the corresponding number in 2050 is projected to rise to 19 million (4.3% of total projected population).

#### Nursing home resident demographic trends

The United States had approximately 15,700 NHs with almost 11,773 (in hundreds) beds and 10,758 (in hundreds) residents in 1973 (17). While the total amount of NHs, beds, and residents decreased from 1999 to 2004, the number of NH beds per 1,000 resident increased from 1,154 in 1999 to 1,593 in 2004 (1, 18). When broken by age groups, the number of elders aged 85 and over [6,745 (51.2%)] has now grown to be the principal group in NHs compared to the 75–84 [4,687 (35.6%)] and 65–74 [1,741 (13.2%)] age groups, respectively (17). Data after 2004 are not available to determine more current trends of NH populations. However, a model utilizing trends in disability and marriage forecasts substantial increases in the incidence of institutionalization among the older adult population within the next decade (19).

#### Health care needs of NH residents

There is evidence that the demand for more healthcare services is growing. As the population ages with increasing lifespan and more effective and efficient health care measures to address acute illnesses, the leading burden of disease shifts to chronic diseases (20). Calkins and his colleagues found that almost 75% of the elderly (age 65 and over) have at least one chronic illness (21). About 50% have at least two chronic illnesses. Chronic circulatory problems, like heart disease, are the number one cause of death among adults over the age of 65 (22).

The large increase in the aging population with chronic diseases is associated with the dramatic changes of dependency ratio and needs for long-term care services (23). Based on the 2004 National NH Survey, more than 98% of NH residents needed help with at least one ADL (Figure 1) (17). In addition, the survey noted that from 1995 through 2004 the percentage of NH residents who needed five ADL services was significantly on the rise. Another study also found that 93.8% of NH residents received help with bathing, 86.5% dressing, 56% toileting, and almost 47% eating (1).

**Figure 1:** **Percentage Distribution of NH Dependencies in Activities of Daily Living (ADL) Dependencies: United States, 1995–2004**. Source: this figure was adapted from data of Center for Disease Control and Prevention (CDC) (17).

Further, the average length of stay since admission was 835 days in 2004 compared to 611 days in 1985 (18, 24), a trend indicating that NH residents consume services for longer periods of time than in prior years. The 4-year period from 1995 to 1999 saw the increasing trends of multiple types of healthcare services including dental services, equipment or devices services, mental health services, and social services for NH residents (1, 25, 26).

### Health care provider: Geriatricians

#### Geriatric medicine workforce: definition and composition

Geriatric medicine was recognized in 1978 as a medical specialty by its special body of knowledge and approach to patient care including the complex medical problems of multiple chronic illness and concurrent acute problems occurring with greater frequency in advanced age (27). For the purpose of this study, “geriatricians” will be the term used to cover physicians that are board-certified in geriatrics and have had prior residency training in internal medicine, family medicine, or general psychiatry (28). Geriatricians have received formal education and training on specific competencies and approaches to elder patient care. Geriatricians are certified through a subspecialty board examination (29–31). The initial board certification of geriatrics (by AMFM and ABIM) started in 1988 (27, 32). All certificates issued in the subspecialties of geriatric medicine and geriatric psychiatry are renewed on a 10 year basis to remain actively certified.

#### Numbers and trends

Trends in the amount and complexity of healthcare services in NH residents are expected to result in a major increased demand for health care workers skilled with and competent to address complex elderly needs. However, current data indicate that the overall number of geriatricians with active certification issued by ABFM, ABIM, and ABPN decreased from 11,184 in 1996 to 8,502 in 2010 (Figure 2) (33–35). With a general population of 40.23 million elders in 2010, this means a board-certified geriatrician to elderly population ratio of 1:5,955 (36). If the geriatric psychiatrists are included, the ratio becomes 1 to 4,736. Several former geriatric-related workforce studies corroborate these findings (37–39).

**Figure 2:** **The Numbers of Active Physicians Certified by American Board of Family Medicine, American Board of Internal Medicine, and American Board of Psychiatry and Neurology from 1992 to 2010**. Source: this figure was adapted from three sources (33–35).

Following earlier higher numbers of first certificates in geriatric medicine (boarded by ABFM, ABIM, or ABPN), the numbers decreased and then leveled off (33–35). While the percentage of first re-certified geriatricians in the three specialty disciplines have remained mainly in the 52–67% range over time (Table 1) (40, 41), the absolute numbers have tended to decline particularly after 2004 - correlating directly to the reduction in the first-certification numbers (33–35).

**Table 1:** **First recertification rates (%) by year and by original certification**.

Year of first certificate (year of first recertification)	ABPN		ABFM		ABIM	
	Certified number	Re-certified number (%)	Certified number	Re-certified number (%)	Certified number	Re-certified number (%)
1990 (2000)	490	329 (67)	473	317 (67)	1,204	550 (46)
1992 (2002)	359	216 (60)	597	372 (62)	1,254	636 (51)
1994 (2004)	422	219 (52)	771	410 (53)	1,568	763 (49)
1996 (2006)	713	275 (39)	254	123 (48)	291	166 (57)
1998 (2008)	65	37 (57)	102	45 (44)	337	215 (64)
2000 (2010)	83	47 (57)	27	21 (78)	200	111 (56)

*This table was adapted from two sources (40, 41)*.

*ABPN, American Board of Psychiatry and Neurology; AMFM, American Board of Family Medicine; ABIM, American Board of Internal Medicine*.

#### Pipeline

Leigh and colleagues pointed out that geriatricians have the highest job satisfaction rating among all specialties (42). However, in the 2006 Medical School Graduation Questionnaire (GQ) report, only 12% of 11,471 students were planning additional training in geriatrics (43). In the 2007 report, about 35% of 12,511 students thought that geriatric/gerontology education was not part of a required course but a separate elective course (44). From 2001 to 2007, increasing numbers of students reported that they were not well prepared to care for older adult patients in long-term health care settings. In the 2010 Medical School GQ report, 16.5% of 13,422 students thought the instruction about care of geriatric patients was inappropriate, 17.8% were dissatisfied with their received education about end-of-life care, and 35.0% even reported their rehabilitative care education was insufficient (45).

Seventeen of 161 allopathic and osteopathic medical schools in the US have departments of geriatrics (46–48). By comparison, every medical school in the UK has a department of geriatrics medicine (9). Based on the American Geriatrics Society, only 0.8% residents in internal medicine or family medicine who graduated from US medical schools (USMDs) entered geriatric medicine fellowship program in 2010 (41). Furthermore, the numbers of geriatrics fellows in three health specialties are not increasing significantly (Figure 3) (49–51). Medical schools with a department of internal medicine trained 327 geriatric medicine fellows in 2002 but only 237 in 2010. The number of geriatric fellows with psychiatry training has also declined from 98 in 1999 to 41 in 2010. Minimal decreases were also noted in the number of geriatric fellows with family medicine background. The numbers of fellowship programs offered by each of these three professional boards have shown very minor increases over the period between 1995 and 2010 (49–51). In contrast, the proportion of international medical graduates (IMGs) in geriatrician fellowship positions (both family medicine and internal medicine) has been increasing over recent decades (52).

**Figure 3:** **Numbers of Geriatric Medicine Fellows between 1995/96 and 2010/11**. Source: this figure was adapted from three sources (49–51).

Lower compensation received by geriatricians may also exacerbate pipeline barriers (53). In general, geriatricians whether in private practice or in academia, receive significantly lower compensation compared to other specialty fields (54). For example, the median salary for a geriatrician in private practice in 2010 was $183,523 compared to over $200,000 for general internists, over $225,000 for rheumatologists, and $240,000 for neurologists (55). Moreover, the pay scales at NHs allowed within the limitations of Medicare and Medicaid reimbursement are quite low among a variety of long-term care settings while the work is emotionally and physically demanding (56, 57). Although geriatricians spent the largest proportion of time (27%) in the NH compared to family physicians (7%) and general internists (6%) the compensation for a geriatrician is less than the other medical fields (58, 59). NH geriatricians have annual salaries at about $160,000 on average (60).

#### Additional perceived barriers to practice and education at nursing homes

Barriers for geriatricians to practice in NHs as evaluated by a group of medical directors are inadequate accessibility to residents’ information, inaccurate medicine-related operations and information gathering, and insufficient nursing support (61). Others include a high volume of non-reimbursable activities, excessive regulations, and heavy paperwork (10, 62, 63). The Institute of Medicine found that the main obstacle to expanding training at non-hospital sites such as NHs is a lack of funding to cover the expenses of residents (8).

## Discussion

The principal findings in this study indicate a worrisome current and projected decline of the geriatrician workforce in the face of a dramatically increasing number of the elderly and their attendant increased burden of chronic and complex diseases. The aging population has been dramatically growing in the past few decades, with an estimated doubling by 2030 compared to 2000. The oldest old (i.e., ages 85 and older) population has now become the fastest growing elder age group in general and the largest age group in NHs (16, 17). These demographic changes result directly in a major demand for expanded health care and public health services, particularly in relation to a high burden of chronic health conditions and comorbidities. The oldest old especially require more intense health services that cannot be managed effectively in their own home or family (64, 65). Dependencies with activities of daily living, long-term care services, mental health, preventive, and social services for NH residents in general are also on the rise (1, 17, 23). It appears a small decrease followed by a leveling off numbers of the NHs, beds, and residents occurred in 2004. More recent data are not available. An explanation for this apparent decline could be related to the preference and availability of other options as home care and assisted living facilities. Regardless, modeling studies project that a greater institutionalization in NHs is anticipated for the future (19, 66).

There is a growing evidence that the capacity of the geriatrician workforce is not keeping up with the health care needs of the aging populations, particularly those in NHs (11, 12, 67). The current ratio (1: 4,736) of geriatricians and geriatric psychiatrists to population aged 65 and older is predicted to decline to 1:7,194 by 2030 (16, 33–35). To retain this current proportion of one geriatrician to 4,736 elders, 6,729 more geriatricians and geriatric psychiatrists need to be trained. This is a major challenge in view of existing trends.

There is also evidence indicating a major shortage of active geriatricians (i.e., currently certified geriatricians) as well as evidence of an increasing number of inactive geriatricians (previously but not currently certified or recertified geriatricians) (68–70). This latter phenomenon appears to be related more to the reduced pool of new certified geriatricians but could also be related to a disinterest in continuing certification due to poor compensation or working conditions (39–41, 56, 59, 71). Further, a number of barriers exist at the student, resident, and fellowship levels that prevent the development of an adequate pipeline of future geriatricians. This pipeline problem is of major concern because it prevents the new geriatricians from adequately replacing those retiring or otherwise leaving the workforce.

The present academic institutions have been unable to provide adequate support for teaching geriatrics because of inadequate funding, insufficient faculty, absent or minimal clinical exposure to NH settings, and lack of time in an already busy curriculum - all likely related to a lack of priority for geriatrics (53, 72). The numbers of geriatric medicine fellowship programs offered by ABFM, ABIM, and ABPN have had only minor increases (49–51, 73). Moreover, decreased filling of fellowships have been demonstrated in spite of the success in increasing positions available for these geriatric fellowships (74). Other contributors to the inadequate pipeline include lower compensation received geriatricians and lower reimbursement from Medicare and Medicaid for geriatric services (53, 54, 58, 60).

This literature search did not find data on the number of geriatricians that were dually board-certified in preventive medicine. While the interpretation of this is not clear, it more probably indicates a small number. It would be optimal to have a geriatric workforce that also had an adequate understanding of public health issues and perspectives, in addition to personal health care.

Taking into account current training numbers, certification and recertification rates, pipelines, and overall decreasing trend of physicians entering the field, the geriatrician workforce is in a state of crisis (40, 41). This has a significance implication for the health of older adults. O’Neill and Barry have pointed out that even if all medical students who graduate each year start to receive geriatrics training today, it would take more than 40 years before the entire physician workforce is prepared sufficiently to meet the unique healthcare needs of the aging population (9).

While this study focused on the geriatric workforce, the authors recognize the importance of other health professional disciplines (e.g., non-geriatrician physicians, nurses, dentists, and pharmacists among others) in providing health care for the elderly. In addition, geriatricians can play important roles as key leaders of change and promote partnering with other health care professionals to enhance geriatric care. Models of best practices by interdisciplinary teams should evolve to improve the coordination of preventive and health care services for older adult populations.

## Conclusion

This study updates and expands findings on the insufficient and diminishing geriatrician workforce in the face of a growing older population with increased disease burden, frailty, and functional dependency. Trends of a deteriorating pipeline of future certified geriatricians portends a serious access problem to geriatricians, health professionals with skills and training in care for older adults. Barriers to overcome in the educational process include inadequate support for faculty, curricula, and teaching venues at academic centers. Disproportionately low compensation for geriatric services and practice compared to other specialties must be addressed to garner medical students’ interest in geriatric medicine and in certified geriatricians’ willingness to maintain their certification. Incentives for future geriatricians could also include forgiveness of medical schools loans, scholarships for continuing education, development of NH specialist culture, and improvement of organizational efficiencies (8, 10, 57, 75, 76).

Although the study focused on NH residents and the geriatrician workforce the findings could be extended to the older adults living in other settings and to other health disciplines involved in geriatric care. Robust interdisciplinary teams commonly headed by geriatricians could advance the appropriate coordination of geriatric services. All medical students or, even better, all health professionals-in-training should receive at a minimum a basic understanding and experience with the care of older adults and their families. While the NH setting should be a principal locus of health professions education, other settings (e.g., assisted living facilities, home care) where older adults live should also be included. Moreover, health services research in quality, cost effectiveness, and access are needed to monitor carefully the capacity and demand for geriatricians. Further, the geriatrician community could take a leadership role in improving the public health system in promoting health and preventing disease among the rapidly growing, frail, older population.

## Conflict of Interest Statement

The authors declare that the research was conducted in the absence of any commercial or financial relationships that could be construed as a potential conflict of interest.

## References

[1] JonesA The National Nursing Home Survey: 1999 summary. Vital Health Stat (2002) 152:1–11612071118

[2] RhoadesJAKraussNA Chartbook #3: Nursing Home Trends, 1987 and 1996. (1999). Available from: http://meps.ahrq.gov/data_files/publications/cb3/cb3.shtml

[3] KasperJO’MalleyM Changes in Characteristics, Needs, and Payment for Elderly Nursing Home Residents: 1999 to 2004. (2007). Available from: http://www.kff.org/medicaid/upload/7663.pdf

[4] WienerJMFreimanMPBrownD Nursing Home Care Quality: Twenty Years After the Omnibus Budget Reconciliation Act of 1987. Washington, DC: The Henry J. Kaiser Family Foundation (2007).

[5] BorgerCSmithSTrufferCKeehanSSiskoAPoisalJ Health spending projections through 2015: changes on the horizon. Health Aff (2006) 25(2):w61–7310.1377/hlthaff.25.w6116495287

[6] Center for Health Workforce Studies (CHWS) The Impact of the Aging Population on the Health Workforce in the United States: Summary of Key Findings. NY: School of Public Health, University at Albany (2006).

[7] FriedLPHallWJ Leading on behalf of an aging society. J Am Geriatr Soc (2008) 56(10):1791–510.1111/j.1532-5415.2008.01939.x19054197

[8] Institute of Medicine (IOM) Retooling for an Aging America: Building the Health Care Workforce. Washington, DC: The National Academies Press (2008).25009893

[9] O’NeillGBarryPP Training physicians in geriatric care: responding to critical need. Public Policy Aging Rep (2003) 13(2):17–21

[10] KatzPRKaruzaJIntratorOVincentM Nursing home physician specialists: a response to the workforce crisis in long-term care. Ann Intern Med (2009) 150(6):411–310.7326/0003-4819-150-6-200903170-0001019293074PMC4756641

[11] BesdineRBoultCBrangmanSColemanEAFriedLPGeretyM Caring for older Americans: the future of geriatric medicine. J Am Geriatr Soc (2005) 53(6):S245–5610.1111/j.1532-5415.2005.53350.x15963180

[12] KaneRLOuslanderJGAbrassIBResnickB Essentials of Clinical Geriatrics, 6th ed. New York: McGraw-Hill (2009). 491 p.

[13] McNabneyMKWillgingPRFriedLPDursoSC The “continuum of care” for older adults: design and evaluation of an educational series. J Am Geriatr Soc (2009) 57(6):1088–9510.1111/j.1532-5415.2009.02275.x19507299

[14] Population Division of U.S. Census Bureau 1990 Census of Population General Population Characteristics. (1990). Available from: http://www.census.gov/prod/cen1990/cp1/cp-1.html

[15] Population Division of U.S. Census Bureau Total Population by Age and Sex for the United States: 2000. (2000). Available from: http://www.census.gov/population/www/cen2000/briefs/phc-t8/index.html

[16] Population Division of U.S. Census Bureau Projections and Distribution of the Total Population by Age for the United States: 2010 to 2050. (2010). Available from: http://www.census.gov/prod/2010pubs/p25-1138.pdf

[17] Center for Disease Control and Prevention (CDC) HHS Gateway to Data and Statistics. (2010). Available from: http://www.hhs-stat.net/scripts/result.cfm?id=NNHS&lk=6

[18] JonesALDwyerLLBercovitzARStrahanGW The National Nursing Home Survey: 2004 overview. Vital Health Stat (2009) 13(167):3–619655659

[19] LakdawallaDGoldmanDPBhattacharyaJHurdMJoyceGFConstantijnWA Forecasting the nursing home population. Med Care (2003) 41(1):8–2010.1097/00005650-200301000-0000312544538

[20] BinstockRHCluffLEMeringOE The Future of Long-Term Care: Social and Policy Issues. Baltimore, MD: The Johns Hopkins University Press (1996).

[21] CalkinsEBoultCWagnerEPacalaJT New Ways to Care for Older People: Building Systems Based on Evidence. New York: Springer (1999).

[22] CDC. Death Rates by Age and Age-Adjusted Death Rates for the 15 Leading Causes of Death in 2006: United States, 1999-2006. (2009). Available from: http://www.disastercenter.com/cdc/Table_9_2006.html

[23] HeinEBloomB Long-term care for the functionally dependent elderly. Am J Public Health (1991) 81(2):223–510.2105/AJPH.81.2.2231899323PMC1404949

[24] HingESekscenskiEStrahanG The National Nursing Home Survey: 1985 summary for the United States. Vital Health Stat (1989) 13(97):1–2492929143

[25] GabrealCJonesA The National Nursing Home Survey: 1995 summary. Vital Health Stat (2000) 13(146):4–3410808755

[26] GabrealCJonesA The National Nursing Home Survey: 1997 summary. Vital Health Stat (2000) 13(147):4–7510957881

[27] MorleyJE A brief history of geriatrics. J Gerontol A Biol Sci Med Sci (2004) 59(11):1132–5210.1093/gerona/59.11.113215602058

[28] Geriatrics Workforce Policy Studies Center (GWPS) Family Medicine, Internal Medicine, and Psychiatry Residency Programs. (2010). Available from: http://www.americangeriatrics.org/files/documents/gwps/Table%204_4.pdf

[29] American Board of Family Medicine (ABFM) Geriatric Medicine: Certification Requirements. (2013). Available from: https://www.theabfm.org/caq/geriatric.aspx

[30] American Board of Internal Medicine (ABIM) Geriatric Medicine. (2013). Available from: http://www.abim.org/specialty/geriatric-medicine.aspx

[31] American Board of Psychiatric and Neurology (ABPN) Information for Applicants. (2011). Available from: http://www.abpn.com/downloads/ifas/IFA_MOC_Geriatric_Psych_MR_NBRD_2011.pdf

[32] BraggEJWarshawGAMeganathanKBrewerDE National survey of geriatric medicine fellowship programs: comparing findings in 2006/07 and 2001/02 from the American Geriatrics Society and Association of Directors of Geriatric Academic Programs Geriatrics Workforce Policy Studies Center. J Am Geriatr Soc (2010) 20(2):169–7810.1111/j.1532-5415.2010.03126.x21039369

[33] GWPS. Comparison of Number of Certificates Awarded to Number of Active Certificates in Geriatric Medicine (Family Medicine). (2011). Available from: http://www.americangeriatrics.org/files/documents/gwps/Figure%201_5.pdf

[34] GWPS. Comparison of Number of Certificates Awarded to Number of Active Certificates in Geriatric Medicine (Internal Medicine). (2011). Available from: http://www.americangeriatrics.org/files/documents/gwps/Figure%201_4.pdf

[35] GWPS. Certifications in Geriatric Medicine and Geriatric Psychiatry Issued by the American Board of Family Medicine, American Board of Internal Medicine, and American Board of Psychiatry and Neurology, 1998-2010. (2011). Available from: http://www.americangeriatrics.org/files/documents/gwps/Table%201_1.pdf

[36] U.S. Census Bureau The Older Population: 2010. (2011). Available from: http://www.census.gov/prod/cen2010/briefs/c2010br-09.pdf

[37] Alliance for Aging Research Medical Never-Never Land: 10 Reasons Why America is Not Ready for the Coming Age Boom. Washington, DC: Alliance for Aging Research (2002).

[38] American Geriatrics Society (AGS) Projected Future Need for Geriatricians. (2012). Available from: http://www.americangeriatrics.org/files/documents/Adv_Resources/GeriShortageProjected2012.pdf

[39] WarshawGABraggEJ The training of geriatricians in the United States: three decades of progress. J Am Geriatr Soc (2003) 51(7 Suppl):S338–4510.1046/j.1365-2389.2003.51345.x12823665

[40] GWPS. Certification and Re-certification in Geriatric Medicine by Year of Original Certification as of 3/11. (2012). Available from: http://www.americangeriatrics.org/files/documents/gwps/Table%201_3.pdf

[41] GWPS. Certification and Re-certification in Geriatric Psychiatry by Year of Original Certification as of 3/11. (2012). Available from: http://www.americangeriatrics.org/…/Ger.Psy.Training.and.Practice.Update.September.2012.pps

[42] LeighJPKravitzRLSchembriMSamuelsSJMobleyS Physician career satisfaction across specialties. Arch Intern Med (2002) 162(14):1577–8410.1001/archinte.162.14.157712123400

[43] Association of American Medical Colleges (AAMC) Medical School Graduation Questionnaire (All Schools Report). Washington, DC: AAMC (2006). 45 p.

[44] AAMC. Medical School Graduation Questionnaire (All Schools Summary Report). Washington, DC: AAMC (2007). 27 p.

[45] AAMC. Medical School Graduation Questionnaire (All Schools Summary Report). (2010). 15 p. Available from: https://www.aamc.org/download/140716/data/2010_gq_all_schools.pdf

[46] GWPS. Departments of Geriatric Medicine. (2011). Available from: http://www.americangeriatrics.org/files/documents/gwps/agp/programs_1.pdf

[47] GWPS. (2012). Academic Geriatric Programs in Allopathic Medical Schools 2010-2011. Available from: http://www.americangeriatrics.org/files/documents/gwps/agp/programs_2.pdf

[48] GWPS. Academic Geriatric Programs in Osteopathic Medical Schools 2010-2011. (2012). Available from: http://www.americangeriatrics.org/files/documents/gwps/agp/programs_3.pdf

[49] GWPS. Family Medicine, Geriatric Medicine Fellowship programs 1991/92-2010/11 [Internet]. (2012) [cited 2012 Aug 20]. Available from: http://www.americangeriatrics.org/files/documents/gwps/Table%203_3.pdf

[50] GWPS. Geriatric Psychiatry Fellowship Programs 1995/96-2010/11. (2012). Available from: http://www.americangeriatrics.org/files/documents/gwps/Table%203_5.pdf

[51] GWPS. Internal Medicine, Geriatric Medicine Fellowship programs 1991/92-2010/11. (2012). Available from: http://www.americangeriatrics.org/files/documents/gwps/Table%203_4.pdf

[52] GWPS. Geriatric Medicine Fellowship Programs, Family Medicine, and Internal Medicine (1st and 2nd Year Fellows, IMGs, and Fellows Completing Program 1991/92-2010/11). (2012). Available from: http://www.americangeriatrics.org/files/documents/gwps/Table%203_2.pdf

[53] GWPS. What Factors are Contributing To – Or are Expected to Contribute To – The Shortage of Geriatricians? (2012). Available from: http://www.americangeriatrics.org/advocacy_public_policy/gwps/gwps_faqs/id:3190

[54] Association of Directors of Geriatric Academic Programs (ADGAP) Geriatricians and compensation. Train Pract Update (2008) 6(1), 1–7

[55] Medical Group Management Association Physician Compensation and Production Survey, 2011 Report Based on 2010 Data. Englewood, CO: Medical Group Management Association (2011).

[56] EvashwickCJ The Continuum of Long-Term Care. New York: Delmar (2001).

[57] Population Reference Bureau (PRB) Aging and the Health Care Workforce. Todays Res Aging (2010) 19, 1–7

[58] American Medical Group Association (AMGA) Physician Compensation Survey. (2012). Available from: http://www.cejkasearch.com/view-compensation-data/physician-compensation-data/#

[59] XakellisGC Who provides care to Medicare beneficiaries and what settings do they use? J Am Board Fam Med (2004) 17(5):384–710.3122/jabfm.17.5.38415355953

[60] HR TrainingCenter.Com Geriatrician Job Description. (2011). Available from: http://www.healthcare-trainingcenter.com/jobs-geriatric.asp

[60] CapiroTVKaruzaJKatzPR Profile of physicians in the nursing home: time perception and barriers to optimal medical practice. J Am Med Dir Assoc (2009) 10(2): 93–710.1016/j.jamda.2008.07.00719187876

[62] LevyCEpsteinALandryL-AKramerA Physician Practices in Nursing Homes: Final Report. Washington, DC: Office of Disability, Aging and Long-Term Care Policy (2006).

[63] LevyCPalatS-ITKramerAM Physician practice patterns in nursing homes. J Am Med Dir Assoc (2007) 8(9):558–6710.1016/j.jamda.2007.06.01517998111

[64] FederJKomisaHLNiefeldM Long-term care in the United States: an overview. Health Aff (2000) 19(3):40–5610.1377/hlthaff.19.3.4010812780

[65] Institute of the Future Health and Health Care 2010: The Forecast, the Challenge. San Francisco: Jossey-Bass Publishers (2000).

[66] SpillmanBCLubitzJ New estimates of lifetime nursing home use: have patterns of use changed? Med Care (2002) 40:965–7510.1097/00005650-200210000-0001312395029

[67] IntratorOCastleNGMorV Facility characteristics associated with hospitalization of nursing home residents: results of a national study. Med Care (1999) 37(3):228–3710.1097/00005650-199903000-0000310098567

[68] Administration on Aging (AoA) Projected Future Growth of the Older Population: By Age 1900-2050. (2011). Available from: http://www.aoa.gov/AoARoot/Aging_Statistics/future_growth/future_growth.aspx#age

[69] JohnsonTD Geriatric work force shortage risks health of aging boomers. Nations Health (2008) 38(5). Available from: http://connection.ebscohost.com/c/articles/32605732/geriatric-work-force-shortage-risks-health-aging-boomers

[70] MitkaM As Americans age, geriatricians go missing. JAMA (2002) 287(14):1792–310.1001/jama.287.14.179211939842

[71] LandefeldCSCallahanCMWoolardN General internal medicine and geriatrics: building a foundation to improve the training of general internists in the care of older adults. Ann Intern Med (2003) 139(7):609–1410.7326/0003-4819-139-7-200310070-0003414530244

[72] EleazerGPDoshiRWielandDBolandRHirthVA Geriatric content in medical school curricula: results of a national survey. J Am Geriatr Soc (2005) 53(1):136–4010.1111/j.1532-5415.2005.53023.x15667390

[73] MoldJWGreenLAFryerGE General internists and family physicians: partners in geriatric medicine? Ann Intern Med (2003) 139(7):594–610.7326/0003-4819-139-7-200310070-0001314530232

[74] Association of Directors of Geriatric Academic Programs (ADGAP) Geriatricians and geriatric psychiatrists. Train Pract Update (2005) 1(2), 1–6

[75] HirthVAEleazerGPDever-BumbaM A Step Toward Solving the Geriatrician Shortage. Williams, MD: The Association of Professors of Medicine (2008).10.1016/j.amjmed.2007.10.03018328311

[76] WarshawGABraggEJThomasDCHoMLBrewerDE Association of Directors of Geriatric Academic Programs. Are internal medicine residency programs adequately preparing physicians to care for the baby boomers? A national survey from the Association of Directors of Geriatric Academic Programs Status of Geriatric Workforce Study. J Am Geriatr Soc (2006) 54(10):1603–910.1111/j.1532-5415.2006.00895.x17038081

